# Low-Dose CT Image Denoising with Improving WGAN and Hybrid Loss Function

**DOI:** 10.1155/2021/2973108

**Published:** 2021-08-26

**Authors:** Zhihua Li, Weili Shi, Qiwei Xing, Yu Miao, Wei He, Huamin Yang, Zhengang Jiang

**Affiliations:** Computer Science and Technology, Changchun University of Science and Technology, Changchun 130022, China

## Abstract

The X-ray radiation from computed tomography (CT) brought us the potential risk. Simply decreasing the dose makes the CT images noisy and diagnostic performance compromised. Here, we develop a novel denoising low-dose CT image method. Our framework is based on an improved generative adversarial network coupling with the hybrid loss function, including the adversarial loss, perceptual loss, sharpness loss, and structural similarity loss. Among the loss function terms, perceptual loss and structural similarity loss are made use of to preserve textural details, and sharpness loss can make reconstruction images clear. The adversarial loss can sharp the boundary regions. The results of experiments show the proposed method can effectively remove noise and artifacts better than the state-of-the-art methods in the aspects of the visual effect, the quantitative measurements, and the texture details.

## 1. Introduction

During recent years, the computed X-ray tomography (CT) has been one of the important practical imaging methods, which has been widely utilized in medical diagnosis. The anatomical structure with high temporal-spatial resolution could be found from CT images, and numerous researchers benefit from CT scans, especially in pathologic diagnosis and treatment domains. However, with the widely use of medical CT, the potential risk of ionizing X-ray radiation to patients has aroused public concern [1, 2].

According to the famous ALARA theory, the minimization of X-ray became one of the research hotspots in CT image fields. Among the many methods, the most popular approach to reduce radiation is reducing X-ray flux by shortening the exposure time and cutting down the operating the X-ray tube current. Unfortunately, the lower the X-ray flux, the noisier the generated CT image. Therefore, one way to address the problem is to reduce the image noise by the algorithm. The common method to reduce noise is filtering. But it is an ill-posed and challenging problem [3–5]. Recently, deep learning techniques have shown their superiority in denoising the image [6–11]. Various denoising models based on convolutional neural networks (CNNs) have been proposed with different network architecture for LDCT denoising [1, 12–14], which include 2D CNNs [2, 12], 3D CNN [1], residual encoder-decoder CNN [13], and cascaded CNN [14]. Besides, different loss functions, such as the mean squared error (MSE) [1, 12–14], adversarial loss [1, 2], and perceptual loss [2], are presented in the denoising model. Different network architectures and loss function may have a profound impact upon the learning process of the network. According to literature [8], the complexity of the denoising model is determined by the network architecture, and the loss function is related to what the denoising model learns from images and data.

In practice, we found the denoising methods with generative adversarial network could get better results than those with CNNs. However, these methods have difficulties of network training and the gradients disappearance [15]. To solve this problem, here, we propose an improved GAN with the Wasserstein distance (SSWGAN) to reduce the noise of the low-dose CT images. Specifically, denoising low-dose CT images can be looked as a translation of low-dose CT images into normal-dose CT (NDCT) images. Our proposed GAN could estimate the distance of distribution between low-dose CT and normal-dose CT. In the process, the perceptual loss based on VGG could preserve as many image details as possible when suppressing the noise. The SSIM loss preserves the structural and textural details after the denoising process, and L1 loss keeps the sharpness of the denoised image, especially in the low contrast regions. In summary, our contributions are as follows:

- An improved WGAN network is introduced as the denoising model
- A novel hybrid loss function is introduced to enhance the denoising model performance
- Compared with a few latest network models, we found our disadvantages and presented the Q-AE model to improve our generator architecture

## 2. Related Work

### 2.1. LDCT Denoising Methods

Generally, the LDCT denoising methods can be divided into three classes:

- *Projection Filtering* [16–18]. Their advantage is the higher computation efficiency. However, they always result in the loss of spatial resolution and edge blur in images
- *Iteration Reconstruction* [19–25]. They outperform in increasing the signal to noise ratio, but they need more computing resources and the accuracy model of the noises
- *Postprocessing* [26–28]. They can be performed on the images directly and have the lower calculating costs so that they have been implied in the CT imaging system and analysis system. There are some residual problems in the processed images yet

With the rapid development of deep learning techniques, associated denoising models have achieved an impressive performance of denoising LDCT images [29, 30]. The learning process includes two major components: network architecture and loss function. The architecture determines the complexity of the denoising model and the loss function controls what the denoising model learn. Recently, lots of methods were proposed. Yi et.al [31] summarized these methods and made a comprehensive comparison. Next, we mainly described the approaches with novel network architecture and the ones with improved loss function,

1. *Network Architecture*. Chen et al. [32] first proposed the low-dose CT image denoising method based on convolution neural network (CNN), who obtained better effects in visual sense and measurements. Then, Chen et al. [13] improved the network structure and they developed a residual encoder CNN (RED-CNN). The results were better than the original CNN. However, their network was complex and time-consuming. To overcome the disadvantages of RED-CNN, Zhang et al. [33] proposed a novel network. Compared with RED-CNN, there were less parameters in their network and their results were better
2. *Loss Function*. Minimizing the MSE based on the difference between the denoised images and the NDCT easily led to overblurred [1, 2], which was proved to correlate poorly with the human perception of image quality [34, 35]. According to literature [8], the optimal MSE estimator suffered from the regression-to-mean problem, which made denoised LDCT look oversmoothed, unnatural, and implausible. The adversarial loss (AL) could result in a sharp image locally indistinguishable from the NDCT image but it does not exactly correspond to the NDCT image globally [36] since the AL optimizes the distance between distributions of the denoised results and NDCT images. Later, many methods presented the perceptual loss (PL) to make denoised images look more similar to NDCT images in the high-level feature space [2]. However, there are other features to be applied in the images, such as the sharpness and structural similarity index. Here, we extend the wise-used hybrid loss function including AL and PL. Our proposed hybrid loss function includes four terms: AL, PL, sharpness loss, and similarity loss to enhance the denoising performance more effectively

### 2.2. Wasserstein GAN Framework

Recently, the GAN [34] architecture was developed as a novel way to model the distribution of the given data. But it has the difficulties of network training and the gradient disappearance [8]. To deal with these limitations, the GAN with the Wasserstein distance (WGAN) was widely used [37, 38], which made use of the Wasserstein distance as the measurement of the difference between the distribution loss and perceptual loss [37]. Besides, gradient penalty was employed as a regular accelerated method for training network (WGAN-GP) [39]. It was important that WGAN-VGG [40] was an approach for low-dose CT, which achieved promising denoised CT images [41], and the perceptual loss was utilized by VGG [41] that pretrained on natural images. WGAN-VGG could overcome the problem of image overblur. Also, SMGAN [42] combined the L1 loss and the multiscale structure loss so that it outperformed the WGAN-VGG in convergence accuracy [40]. But sometimes, the reconstruction images were fuzzy. Besides, the gradient penalty term weakened the express ability of GAN [43]. Furthermore, researchers found the denoising model without deconvolutional layers, which is the transpose of convolutional layers [44], implies that the input and the output of the denoising model may have different sizes. To keep the size of denoised CT images equal to that of the input, U-net architecture are used in denoising LDCT images [45–51]. Shan et al. [8] proposed the conveying path-based convolutional U-net denoising model, which is called as CPCE. Fan et al. [15] improved the method and proposed a denoising framework, who replaced the inner product in current artificial neurons with a quadratic operation on input data. Their method is called the Q-AE.

## 3. Denoising Framework

### 3.1. Principle and Model of Denoising

Generally, the noise distribution in CT images is treated as the combination of quantum Poisson and electronic Gaussian noise. But the noise in reconstruction images is complex, and its distribution is always nonuniform. Besides, the relationship between NDCT and LDCT cannot be described with an accuracy mathematical model. So only with conventional methods, we could hardly obtain better results of denoising LDCT images. Fortunately, the uncertain noise model can be estimated by deep learning techniques, because of its strong ability of capturing features.

Denoising LDCT images can be represented as the below model. Assume that $x\in R^{N\times N}$ represents the NDCT image and $y\in R^{N\times N}$ represents the corresponding LDCT, our goal is to confirm a function G which maps **y** to **x**:

(1) $$\begin{array}{c} G:y⟶x. \end{array}$$

The generative and adversarial abilities of GAN can be applied to extract features from deep levels with the spatial information of reconstruction images, so that GAN can identify the noise and effective image details. GAN usually includes a pair of neural networks: a generator *G* and a discriminator *D* [52, 53]. The generator *G* can learn the real distribution of NDCT, and the discriminator *D* can make the best effort to distinguish between real or fake samples generated by *G*. This pair of networks is often trained alternatively, so the competition encourages the generated samples to be hardly distinguished from real ones. Finally, we could obtain CT images of better quality.

### 3.2. The Structure of our GAN

Mathematically, *G* and *D* could be formed as a two-role minimax game:

(2) $$\begin{array}{c} \begin{array}{c} \text{minmax}\\ G\;D \end{array}E_{x∼P_{\text{data}}\left(x\right)}\left[\log D\left(x\right)\right]+E_{y∼P_{y}\left(y\right)}\left[\log\left(1-D\left(G\left(y\right)\right)\right)\right], \end{array}$$

where *E* represents the expectation value, *P*_data_ and *P*_*y*_ represent real and noise distributions, respectively. In the regular GAN, the Jensen-Shannon (JS) divergence is utilized to compute the similarity of two kinds of data distribution [54]. But, as mentioned above, the JS divergence easily results in gradient vanishing. Here, we adopt the Wasserstein distance [38] instead of JS divergence to ensure the training stability of the neural network. The main structure of our network is shown in Figure 1. As shown in the figure, there are four parts in our SSWGAN network, which is the generator, discriminator, sharpness detection network, and hybrid loss function, respectively.

#### 3.2.1. The Architecture of our Generator

As shown in Figure 2, the proposed generator *G* is different from the traditional noise reduction models. Here, we utilize the ADNet [55] with 17 layers as our generator. There are four parts in our generator network, which represents sparse block (SB), feature enhance block (FEB), attention block (AB), and reconstruction block (RB), respectively. In particular, SB could reduce noise with dilated and common convolution to achieve the optimal balance between performance and efficiency. FEB combines the global and local feature information to improve the representation ability of models. AB is often applied to extract the implied noise in the complex background accurately. Utilizing both FEB and AB could both improve the efficiency and reduce the complexity of training the network model. RB generates the NDCT images of better quality with the obtained noise map and given LDCT images.

#### 3.2.2. The Architecture of our Discriminator

As shown in Figure 3, the input of the discriminator is the NDCT generated by *G* and the real NDCT. Our discriminator *D* is designed to distinguish the real one from the two NDCT images. The discriminator includes 6 convolution layers and 3 full-connected layers. Among the convolution layers, there are 64 filters in the first two layers, 128 filters in the middle two layers, and 256 filters in the final two layers. After each convolution operation, there is an activation function ReLU [56]. The step size of convolution is 1 and the filter size is 3 × 3. The end of the discriminator is fully-connected layers, and there are 1024 outputs, 512 outputs, and 1 output, respectively. With the discriminator, we could obtain the difference of the generated NDCT and real NDCT.

#### 3.2.3. Sharpness Detection Network

Numerous noise reduction methods are poor in fuzzy edge. Traditional nonlinear optimization algorithms are to average adjacent pixels or utilize the self-similar patch. However, when the noise level is high, these optimization algorithms are not efficient because of the high similarity between noise and edge. Although the discriminator of GAN could output more clear images and distinguished images from the candidates, it is not efficient in the low contrast regions because the antagonism loss used in GAN could not ensure that the images are able to be reconstructed accurately.

Recently, a few more flexible and complex methods were proposed, which mainly made use of the statistical differences of the specific properties between the fuzzy regions and the sharp regions, such as the gradient information [57] and discrete cosine coefficient [58]. Other methods utilized the sparse coding way to decompose local paths and obtained sharper images by quantifying the local sharpness. Also, the other methods could generate sharp images, for example, the one based on depth map estimation [59]. It is hard to make a mark in the low contrast regions of medical images, so we introduce a sharpness detection network, represented by *S*, and use the method proposed by Yi and Eramian [60] because of its strong sensitivity in low contrast regions. When implementing SSWGAN, we transfer the NDCT results generated by *G* to the sharpness detection network *S* and compare the sharpness images of our generated results with the images of real ones. Because the sharpness images are shown with grayscale, the pixel values represent the local sharpness. With the sharpness images, we can calculate the mean square error between the two sharpness images and update the weight of network according to the calculated results.

#### 3.2.4. Hybrid Loss Function

The main challenge of the training network is to preserve as much texture detail as possible when reducing noise. The hybrid loss function can keep the training process of SSWGAN within bounds. With the hybrid loss function, the differences between the generated NDCT images and real NDCT images can be measured and the weights of generator *G* can be updated by back propagation (BP). In order to improve the denoising network, our hybrid loss function includes four parts, which is adversarial loss, perceptual loss, sharpness loss, and structural similarity loss, respectively.

*(1) Adversarial Loss*. As described in Ref [2], minimizing the least-squares loss could approximate the distribution of LDCT according to the NDCT, and finally, we could obtain better denoised images. However, it does not match well the corresponding NDCT in detail. Here, we introduce the adversarial loss to let our *G* generate denoised CT images as real as possible. Adversarial loss could be described as follows:

(3) $$\begin{array}{c} L_{\text{WGAN}}\left(G,D\right)=-E_{x}\left[D\left(x\right)\right]+E_{z}\left[D\left(G\left(z\right)\right)\right]+\lambda E_{\hat{x}}\left[{\left({\left\|\nabla_{\hat{x}}D\left(\hat{x}\right)\right\|}_{2}-1\right)}^{2}\right]. \end{array}$$

Here, the first two items represent the Wasserstein distance, and the final item represents the gradient vanish one utilized for network normalization. *G* and *D* are the generator and discriminator. **E** is a set of data samples with specific distribution. $\hat{x}$ is the generated NDCT image, and *λ* is the penalty coefficient. Minimize adversarial loss can keep more texture details.

*(2) Perceptual Loss*. The most important for medical images is to keep the necessary features used in pathologic diagnosis [61]. Mean squared error (MSE) is always utilized as the loss function, which can result in images aliasing and details lost. Perceptual loss can calculate the distance between the generated images and the real images in the feature space of human perception instead of the distance in pixel space. With the perceptual loss, the generated denoised NDCT images could preserve the origin feature in real NDCT images, which is not achieved with other loss function. The perceptual loss can be described as follows:

(4) $$\begin{array}{c} L_{\text{Perceptual}}\left(G\right)=E_{\left(x,y\right)}\left[\frac{1}{whd}{\left\|\phi \left(G\left(y\right)\right)-\phi \left(x\right)\right\|}_{F}^{2}\right], \end{array}$$

where *ϕ* is the feature extractor, and ‖·‖_*F*_ is the Frobenius norm. Here, we adopt the pretrained VGG-19 network [41] as the extractor, *w*, *h*, *d* represent the width, height, and depth, respectively. Because VGG-19 takes the color images as the input and CT images are often in grey scale, we convert the CT images into RGB channel as the input of VGG-19. There are 16 convolution layers and 3 full-connected layers in VGG-19. Among the convolution layers, the output of the 16th layer is the extracted feature of VGG and is used as the loss function:

(5) $$\begin{array}{c} L_{\text{VGG}}\left(G\right)=E_{\left(x,y\right)}\left[\frac{1}{whd}{\left\|\text{VGG}\left(G\left(y\right)\right)-\text{VGG}\left(x\right)\right\|}_{F}^{2}\right]. \end{array}$$

*(3) Sharpness Loss*. Here, we propose a sharpness loss used in sharpness detection network to evaluate the sharpness of images. The generator *G* is asked to not only generate the image as similar to the real one as possible but also generate the clear image as close to the real image as possible. The sharpness loss is described in mathematical form:

(6) $$\begin{array}{c} L_{\text{Sharp}}\left(G\right)=E_{\left(x,y\right)}\left[{\left\|S\left(G\left(y\right)\right)-S\left(x\right)\right\|}_{2}\right], \end{array}$$

where ‖·‖_2_ is *L*_2_ distance.

*(4) Similarity Loss*. In medical CT images of different dose levels, the feature correlation is usually strong. Structural similarity index (SSIM) includes three parts, which is luminance, contrast, and structure. SSIM is a better evaluating indicator than MSE and peak signal-to-noise ratio (PSNR) in visual tasks. To measure the similarity between denoised CT images and normal-dose version, the SSIM can be described:

(7) $$\begin{array}{c} \text{SSIM}\left(x,y\right)=\frac{2\mu_{x}\mu_{y}+C_{1}}{\mu_{x}^{2}+\mu_{y}^{2}+C_{1}}*\frac{2\sigma_{x}\sigma_{y}+C_{2}}{\sigma_{x}^{2}+\sigma_{y}^{2}+C_{2}}*\frac{\sigma_{xy}+C_{3}}{\sigma_{x}\sigma_{y}+C_{3}}, \end{array}$$

where *μ*_*x*_, *μ*_*y*_, *σ*_*x*_, *σ*_*y*_, and *σ*_*xy*_ represent the means, standard deviations, and the cross-correlation of two images, respectively, and *C*_1_, *C*_2_, and *C*_3_ are the constants. Besides, when **x** and **y** are more similar, the value of SSIM is closer to 1. Thus, we set the loss function for SSIM as follows:

(8) $$\begin{array}{c} L_{\text{SSIM}}\left(G\right)=1-\text{SSIM}\left(x,y\right). \end{array}$$

It is worth noting that the SSIM loss can be back-propagated to update the parameters of our network, when giving its property of differentiability. Here, we make use of SSIM to calculate the overall similarity between the NDCT images and LDCT images.

In summary, the overall objective function of our adapted SSWGAN is represented as follows:

(9) $$\begin{array}{c} L_{\text{SSWGAN}}=\alpha L_{\text{WGAN}}\left(G,D\right)+\beta L_{\text{perceptual}}\left(G\right)+\gamma L_{\text{Sharp}}\left(G\right)+\omega L_{\text{SSIM}}\left(G\right), \end{array}$$

where *α*, *β*, *γ*, and *ω* are weight coefficients of the above four terms.

## 4. Results and Discussion

### 4.1. Dataset for Experiments

To show the capacity of our proposed denoising SSWGAN for LDCT image, four real clinical CT image datasets were applied in our study in order to avoid overfitting problem. The four datasets were MDLCT dataset authorized by Mayo Clinic for “2016 NIH-AAPM-Mayo Clinic Low Dose CT Grand Challenge,” the lung CT image dataset [62], the real piglet CT image dataset [63], and the thoracic CT image dataset [64].

The MDLCT dataset includes 2378 NDCT images and the corresponding simulated LDCT (quarter dose) from ten anonymous patients [12]. The matrix of each CT images is 512 × 512, and the thickness is 3.0 mm. Inspired by Ref. [57], we divided the dataset into two groups. One of the groups includes 2168 paired images from nine patients used in the training process. The other one contains 210 paired images from the last patient utilized as the test dataset. During the training stage, we extracted the patches whose size was 55 × 55. Totally, we extracted approximately 106 paired patches used for capturing local details instead of wasting huge memories, which improved the efficiency of the training.

The lung CT images dataset is created from a patient with the method proposed in Ref. [64], including 663 slices. The CT scans of the patient are from The Cancer Imaging Archive (TCIA). The piglet CT image dataset contains 900 images with 100 KVp, 0.625 mm thickness. The thoracic CT image dataset includes 407 pairs of CT images from an anthropomorphic thoracic phantom. The current tube for NDCT and LDCT images is 480 m As and 60 m As, respectively, with a peak voltage of 120 KVp and slice thickness of 0.75 mm. We randomly selected 30% of images using in the test stage, and the size of each image is 512 × 512.

### 4.2. Parameter Setting

Our framework is implemented within Python's platform, Pytorch, and TensorFlow. All experiments run on a personal computer (Intel i5 7400 with 16 G random memory) and accelerated by a NVDIA RTX 2080 GPU with 16 G memory.

The generator and discriminator of our SSWGAN are both optimized utilizing the adaptive momentum estimation (Adam) proposed in Ref. [65]. The size of our mini-batch is 96. The learning rate is set to 10^−3^ used for training 100 epochs and set to 10^−4^ used for training 100 epochs. The coefficients of our hybrid loss function are set *α* = 0.005, *β* = 0.0995, *γ* = 0.95, *ω* = 0.95, and *λ* = 10, respectively. As shown in Figure 4, our network can be convergent after training 100 epochs.

### 4.3. Image Evaluation Criteria

To evaluate the quality of generated images, we adopt three objective evaluation criteria, which are PSNR [12], SSIM [35], and feature similarity index (FSIM) [66]. PSNR calculates the average pixel difference between the generated NDCT images and real NDCT images, which is used for evaluating the denoising ability of different methods. SSIM calculates the structural difference between the generated NDCT images and real NDCT images, which is used for evaluating the similarity of two images. FSIM calculates the feature difference between the two images, which represents the feature-preserving ability of different methods.

## 5. Experimental Results and Discussion

Note that, we describe the advantages of our algorithm framework in two ways: (1) compared with other widely used traditional LDCT denoising methods and (2) compared with the latest LDCT denoising methods based on GAN.

### 5.1. The Comparison between Ours and the Traditional LDCT Denoising Algorithms

To demonstrate, our proposed method has advantages in denoising LDCT images, and we compare ours with other widely used traditional LDCT denoising methods including BM3D [67], CNN200 [12], WGAN [2], and SMGAN [42]. Among these methods, BM3D is one of the most popular traditional approaches utilized for denoising LDCT images. CNN200, WGAN, and SMGAN are three representative denoising methods based on CNN. CNN200 adopts the encoder-decoder convolutional neural network with MSE loss. WGAN and SMGAN make use of Wasserstein distance and sharing similar network architecture. But their loss function is different between each other.

Figure 5 gives the visual results for the MDLCT dataset. As shown in Figure 5, there are much noise in LDCT images, which results in the blurred images and hard to distinguish the structure and details of images. The corresponding NDCT image is much clearer and of better quality in comparison. The third subgraph is the denoising result of BM3D, where there is a small part of noise. Affected by significant blocky, some edges and small structures are too blurred. The fourth subgraph shows the result of CNN200. From the fourth image, it can be found that this method suppresses noise to some degree; however, there are still some noise and artifacts in the images which are after denoising. From the fifth image and sixth image, the denoising methods based on GAN not only reduce most noise and artifacts but also preserve structural details. Compared with the fourth image, there are less noise in the fifth one. But some edge details are loss. The sixth subgraph is the result of SMGAN. It can be seen that SMGAN smoothens the images excessively, and some crucial structures, like the region of porta, are over blurred. From the right image, it can be seen that our framework outperforms in the content details and textural information than the other methods.

As shown in Figures 6–8, all images are denoised results of the above methods based on lung CT images dataset, piglet CT images dataset, and thoracic CT images dataset. We can obtain the same conclusion from the comparison of all methods in Figures 6–8 as the one in Figure 5. Our method could perform better in reducing artifacts and noise. Our denoised images are closer to the real NDCT images.

We computed the SSIM, FSIM, and PSNR of all denoised images. The results are listed in Tables 1–4, respectively. Here, we evaluated the average values of the dataset.

In Table 1, the results are calculated for the images of the MDLCT dataset. Our framework obtains the best results in aspects of SSIM, PSNR, and FSIM. Our PSNR value is averagely 2.7287 dB higher than other methods, the SSIM of our framework is averagely 0.0385 higher than others, and our FSIM result is averagely 0.0414 higher than others. The result of Table 1 shows that our framework gains the best results in respect of all quantitative measurements. From Tables 2–4, we can get the same conclusion, that is to say, it is important to point out that our statistical value is nearest to that of the NDCT images and obtained the best matching textural statistics to NDCT image than other methods.

Besides, to exhibit that our framework has the advantage in terms of convergence, taking results of the MDLCT dataset as an example, we evaluated the quantitative measurements 1-SSIM (the smaller the values, the better the image is) during the training process of different methods. The results can be seen in Figure 9.

As shown in Figure 9, WGAN-VGG and WGAN-MSE are convergent at the point, where the epoch number is 60. CNN200 and SMGAN could achieve convergence at the point, where the epoch number is 45. Our framework can be convergent at the point where the epoch number equals 30. The efficiency of our method is higher than other methods, and it can be seen in Figure 9 that our images under convergence are of better quality.

### 5.2. The Comparison between Ours and the Latest LDCT Denoising Algorithms Based on GAN

To compare with the latest LDCT denoising algorithms based on GAN including the CPCE algorithm [8] and the Q-AE algorithm [15], we conduct experiments on the MDLCT dataset.  Figure 10 shows the results.

Seen from the above figure, we found both of the algorithms perform better than ours. Our image suffers from the oversmoothed details and the loss of texture information (indicated by red arrow and green arrow). The quantitative results can be seen in Table 5. From the results, our proposed denoising framework is not good as the latest algorithms based on GAN.

To analyse the reason why our algorithm is not so good, we compare our network architecture and loss function with the latest algorithms based on GAN. Then, we found the disadvantages of our proposed framework. First, our generator does not involve the deconvolutional layers. As described in literature [15], it easily implies that the input and the output may have different sizes. More seriously, the texture is lost. Then, the convolutional layers do not preserve enough features. To overcome these shortcomings, we improve our framework. Inspired by the literature [15], we modified the architecture of our generator, and it can be seen in Figure 11.

Seen from the above figure, we replace our original SSWGAN with (network). We keep our loss function unchanged. After improving our network architecture, we compare the new obtained results with the latest denoising methods. The quantitative results are seen in Table 6. From the results, our improved method outperforms better.

Figure 12 and Table 7 show the quality assessment index of the comparison between our improving result and original result on lung CT images dataset and piglet CT images dataset, including the PSNR, SSIM, and FSIM. The results show that our improvement is better than the originals. This is largely due to that the (network) with Q-AE model could give a high-order nonlinear sparse representation with a reasonable model complexity.

### 5.3. Discussions and Analysis

In our framework, we propose the SSWGAN with hybrid loss function to denoise the LDCT images. Then, inspired by the latest algorithm, we improve our network architecture. The major difference between ours and other methods is the utilization of hybrid loss function except the network architecture. When deep learning approaches are presented in image processing, we can obtain better results than the state-of-the-art LDCT denoising methods because we can capture high-level abstract features from training data. To a large extent, the loss function of deep learning influences the LDCT image restoration process. Here, we compared different loss function performance on LDCT image restoration: (1) only with adversarial loss, (2) only with perceptual loss, (3) only with the sharpness loss, (4) only with the structural similarity loss, and (5) with the hybrid loss. Also, we took the MDLCT dataset as an example. The results were shown in Figure 13.

Seen from Figure 13, the adversarial loss makes the edge sharper (shown as Figure 13(a)). The perceptual loss makes the edge more obvious (shown in Figure 13(b)), and it easily results in the artifacts. The sharpness loss can generate a clear image (shown in Figure 13(c)), however, it losses part of details. The structural similarity loss can preserve more details and image structures while reducing noise. For evaluating the quality of images, we adapt the PSNR, SSIM, and FSIM. The results are shown in Table 8.

From Table 8, we can find that although any one of the four loss functions has advantages, only with one kind of loss function, the quality of image is lower than the image with hybrid loss function. In addition, with hybrid loss function, we could achieve gradient penalty and acceleration of convergence.

Since (parameter) of our hybrid loss function can make impact on the denoising results. Here, we try to find the relationship between our chose parameters and the quality of the denoised images. In order to determine the optimal weighting parameter for each loss item in our hybrid loss function, we often rely on our experimental experience. When we need to select the optimal parameters, first, we fix *β*, *γ*, and *ω* and select the optimal *α*. Then, we fix *α*, *γ*, and *ω* and determine the optimal *β*. The process of determining the optimal *γ* is the same as determined optimal *β*. Finally, we obtain the best value of *ω* based on optimal *α*, *β*, and *γ*. When choosing the value of parameter, we are used to measuring the denoising performance with different values, as shown in Figure 14. Here, we take the parameter *β* as an example and use the MSE as the metric.

The results demonstrate that the chosen parameters have influence on the denoising performance.

## 6. Conclusions

In this paper, we propose a novel framework for denoising low-dose CT images, which utilize noise learning and enhanced a SSWGAN with hybrid loss function, including adversarial loss, perceptual loss, sharpness loss, and structural similarity loss. First, in order to obtain a noise-free CT image, our generator can learn the noise distribution from the LDCT image and then reduce the noise from the input. After training offline with pairs of the low-dose and normal-dose CT images, our method can reduce the noise of original CT images better than the state-of-the-art methods. In the future, we shall improve our network to obtain noise-free CT images of better quality by denoising the low-dose CT images.

## Figures and Tables

**Figure 1:** The framework of our SSWGAN network for denoising LDCT images.

**Figure 2:** The framework of our generator. As shown in the figure, it could learn the noise and then generate the denoised output according to the input LDCT.

**Figure 3:** The framework of our discriminator. As shown in the figure, it could learn to judge that if the input is generated by *G* or a real NDCT image.

**Figure 4:** The training curves for different terms of our loss function, which is generator loss (a), Wasserstein distance (b), and discriminator loss (c).

**Figure 5:** Denoising results of the different algorithm on the MDLCT dataset. From left to right, the subgraph indicates the detail of different images: the low-dose CT (LDCT), normal-dose CT (NDCT), BM3D, CNN200, WGAN, SMGAN, and our framework.

**Figure 6:** Denoising results of the different algorithm on the lung CT images dataset. From left to right, the subgraph indicates the detail of different images: the low-dose CT (LDCT), normal-dose CT (NDCT), BM3D, CNN200, WGAN, SMGAN, and our framework.

**Figure 7:** Denoising results of the different algorithm on the Piglet CT images dataset. From left to right, the subgraph indicates the detail of different images: the low-dose CT (LDCT), normal-dose CT (NDCT), BM3D, CNN200, WGAN, SMGAN, and our framework.

**Figure 8:** Denoising results of the different algorithm on the thoracic CT images dataset. From left to right, the subgraph indicates the detail of different images: the low-dose CT (LDCT), normal-dose CT (NDCT), BM3D, CNN200, WGAN, SMGAN, and our framework.

**Figure 9:** Convergence comparison between our framework and different methods.

**Figure 10:** Denoising results of the different algorithm on the MDLCT dataset. From left to right, the subgraph indicates the detail of different images: our framework, Q-AE, CPCE-3D, and NDCT images.

**Figure 11:** Architecture of our improved generator. Q-Conv indicates the “quadratic convolution” [15], and Q-Deconv indicates the “quadratic deconvolution” [15].

**Figure 12:** Quantitative results of the lung CT images dataset, piglet CT images dataset, and thoracic CT images dataset utilizing our original network and improved network. Seen from the figure, sub-Fig (a) is the PSNR results, sub-Fig (b) is the SSIM results, and sub-Fig (c) is the FSIM results.

**Figure 13:** Denoising comparison between different loss function.

**Figure 14:** The effect of the parameter *β* in our hybrid loss function on the validation set from the MDLCT dataset. Under the detail images, the noise level of each CT image (the difference between each result and the LDCT image). From the left to the mid column ([0, 0.995]), the noise level of CT image gradually decreases as the *β* increases. From the mid column to the right column ([0.995, 3.0]), the noise level of CT image increases as the *β* increases.

**Table 1:** Quantitative results for Figure 5 (the results of MDLCT dataset) utilizing different methods. Low dose indicates the noisy low-dose images, and others are the results of different methods.

Quantitative measurements	LDCT	BM3D	CNN200	WGAN	SMGAN	Ours
PSNR/dB	24.4411	25.4434	27.8083	28.1414	27.5667	28.8961
SSIM	0.7882	0.7937	0.8362	0.8428	0.8394	0.8596
FSIM	0.912	0.9306	0.9675	0.9484	0.9660	0.9762

**Table 2:** Quantitative results for Figure 6 (the results of lung CT images dataset) utilizing different methods. Low dose indicates the noisy low-dose images, and others are the results of different methods.

Quantitative measurements	LDCT	BM3D	CNN200	WGAN	SMGAN	Ours
PSNR/dB	14.5911	24.7603	33.1926	33.7454	34.6880	35.5760
SSIM	0.2008	0.6750	0.8804	0.9281	0.9310	0.9533
FSIM	0.9232	0.9540	0.9683	0.9565	0.9630	0.9769

**Table 3:** Quantitative results for Figure 7 (the results of piglet CT images dataset) utilizing different methods. Low dose indicates the noisy low-dose images, and others are the results of different methods.

Quantitative measurements	LDCT	BM3D	CNN200	WGAN	SMGAN	Ours
PSNR/dB	39.93	41.46	44.18	44.31	44.83	45.10
SSIM	0.9705	0.9733	0.9794	0.9802	0.9816	0.9885
FSIM	0.9155	0.9422	0.9614	0.9550	0.9677	0.9765

**Table 4:** Quantitative results for Figure 8 (the results of thoracic CT images dataset) utilizing different methods. Low dose indicates the noisy low-dose images, and others are the results of different methods.

Quantitative measurements	LDCT	BM3D	CNN200	WGAN	SMGAN	Ours
PSNR/dB	25.66	30.86	33.57	33.60	33.73	34.03
SSIM	0.4485	0.6552	0.8001	0.8018	0.8049	0.8159
FSIM	0.9103	0.9486	0.9630	0.9565	0.9670	0.9744

**Table 5:** Quantitative results for Figure 10 (the results of MDLCT dataset) utilizing different methods. Low dose indicates the noisy low-dose images, and others are the results of different methods.

Quantitative measurements	Ours	Q-AE	CPCE-3D
PSNR/dB	28.8961	32.712	30.137
SSIM	0.8596	0.95266	0.905

**Table 6:** Quantitative results for Figure 10 (the results of MDLCT dataset) utilizing different methods. Low dose indicates the noisy low-dose images, and others are the results of different methods.

Quantitative measurements	Our originals	Q-AE	CPCE-3D	Our improvement
PSNR/dB	28.8961	32.712	30.137	32.848
SSIM	0.8596	0.95266	0.905	0.95649

**Table 7:** Quantitative results for Figure 12 utilizing our original network and improved network. “Ori” indicates the results of our original network, and “Imp” indicates the results of our improved network.

Quantitative measurements	Lung CT images dataset	Piglet CT images dataset	Thoracic CT images dataset
PSNR/dB	(Ori) 35.5760	(Ori) 45.10	(Ori) 34.03
	(Imp) 36.3950	(Imp) 45.962	(Imp) 35.2649
SSIM	(Ori) 0.9533	(Ori) 0.9885	(Ori) 0.8159
	(Imp) 0.9645	(Imp) 0.9892	(Imp) 0.8651
FSIM	(Ori) 0.9769	(Ori) 0.9765	(Ori) 0.9744
	(Imp) 0.9774	(Imp) 0.9767	(Imp) 0.9759

**Table 8:** Quantitative results for Figure 13 (the results of MDLCT dataset) utilizing different loss function.

Quantitative measurements	Adversarial loss	Perceptual loss	Sharpness loss	Structural similarity loss	Hybrid loss
PSNR/dB	24.66	26.86	26.57	25.60	28.8961
SSIM	0.8485	0.7552	0.8301	0.8058	0.8596
FSIM	0.9485	0.9446	0.9635	0.9665	0.9762

## Data Availability

No data were used to support this study.
